# Medical experiences of patients with breast cancer using smart hospital apps: A qualitative study

**DOI:** 10.1016/j.heliyon.2025.e42573

**Published:** 2025-02-12

**Authors:** Xin Peng, Lingling Tang, Ping Gao, Wei Liu

**Affiliations:** a Department of Cancer Center, Union Hospital, Tongji Medical College, Huazhong University of Science and Technology, Jiefang Avenue 1277, Wuhan, 430022, China; b Department of Information and Data Center, Union Hospital, Tongji Medical College, Huazhong University of Science and Technology, Jiefang Avenue 1277, Wuhan, 430022, China

**Keywords:** Smart hospital, Medical experience, Informatization, Artificial intelligence, Qualitative research

## Abstract

**Objective:**

To examine medical experiences of patients with breast cancer with smart hospital apps and their expectations for future development.

**Methods:**

A descriptive qualitative research method was employed to conduct in-depth interviews with 40 patients with breast cancer who used smart hospital apps. Content analysis was performed to analyze and organize the interview data.

**Results:**

Five main themes and two sub-themes were identified. The main themes were as follows: positive experiences with using smart hospital apps, difficulties with data sharing across multiple campuses, interpersonal communication and coping, smart healthcare not a free choice, and expectations for development of smart hospitals. The sub-themes were as follows: precise information delivery mechanisms and intelligent healthcare navigation.

**Conclusion:**

Researchers should enhance communication from the patient's perspective to understand the problems patients encounter when using smart hospitals for medical treatment and their expectations for development of smart hospitals. Efforts should focus on minimizing patient usage barriers and accelerating smart hospital development.

## 1 Introduction

Promoting high-quality development of hospitals has become an intrinsic requirement for public hospital reform in the new era [1,2]. In 2021, the General Office of the State Council issued the "Opinions on Promoting the High-Quality Development of Public Hospitals," which introduced new trends for guiding the development of public hospitals and advancing the construction of smart hospitals. Smart hospitals leverage Internet-based technologies, including cloud computing, IoT, and mobile applications, to enhance hospital informatization and automation. This facilitates more convenient appointment registration, in-clinic settlement, and hospital admission reservations for the public, meeting their healthcare service needs and contributing to healthcare system reform [3]. During the "14th Five-Year Plan" period, promoting the construction of smart hospitals to achieve high-quality development of public hospitals has become a hot topic in hospital management circles. For different groups, a smart hospital has different meanings. A patient experience-based smart hospital emphasizes providing more convenient medical services to patients, including offering the best treatment plans, standardizing medical practices, avoiding excessive medical treatments, and reducing healthcare costs. Despite the potential benefits, patient experiences with intelligent healthcare services remain underexplored.

As smart hospitals in China are still in their early stages, significant challenges persist, including unclear objectives and implementation strategies [4]. Patients, as a special service group, must have their needs recognized [5]. Therefore, conclusions drawn from studies on e-commerce platforms are difficult to apply. Despite the rise of artificial intelligence driving the development of smart hospitals and providing convenience for patients—such as apps allowing patients to view and manage personal health data—currently, this is limited to data from the past three months and lacks guidelines. Patient experience is a key factor in the construction of smart hospitals; however, previous studies have paid little attention to it. The author argues that development of smart hospitals relies not only on technological advancements but also on experiences and expectations of patients during the usage process. Therefore, this study examined the experiences of patients with breast cancer of different ages, educational backgrounds, and disease conditions using smart medical services, based on patient feedback and data analysis. It aimed to explore key issues in smart hospital construction, provide decision-making support for high-quality planning, construction, and development of smart hospitals, enhance patient satisfaction, and promote sustainable development of hospitals. The author's hospital information data center, using the smart hospital grading evaluation standard system as the core, completed the design of an integrated smart hospital architecture, including smart logistics, smart security, smart medical engineering, smart wards, smart outpatient services, and a command and dispatch center. The smart ward system includes health education, questionnaire follow-up, medication check-ins, indicator returns, medical planning, health consultation, follow-up reminders, and anomaly alerts. This study conducted semi-structured interviews with 40 patients with breast cancer regarding their application experiences with the smart hospital system. From the perspective of patients using the smart hospital app for healthcare, this study sought to understand how patients described their experiences with usage. This study aimed to explore the following three research questions: 1. What factors influence patients' positive experiences with the smart hospital app? 2. What factors influence patients' negative experiences with the smart hospital app? 3. What are patients' expectations for future development of smart hospitals? Exploring these questions will provide reference for development of smart hospital construction.

## 2 Objects and methods

### 2.1 Participants

The participants were selected using purposive sampling from the breast tumor department of our hospital between March and June 2023. The inclusion criteria were as follows: ① age ≥18 years; ② meeting the diagnostic criteria for breast cancer; ③ being able to use a smartphone and complete the survey independently or with assistance; ④ no language barriers; ⑤ using the smart hospital app for ≥1 month. The exclusion criteria were as follows: ① other concurrent malignant tumors; ② patients with mental disorders or cognitive impairments. To enhance representativeness of the respondents, we considered factors such as age, gender, type of disease, and education level and incorporated a diverse range of respondents. The sample size was determined based on the principle of information saturation, with no new topics introduced during the interviews. A total of 40 patients with cancer were interviewed. Participants’ characteristics are shown in Table 1.

**Table 1:** General information of participants.

Participants' Characteristics	Numbers
**Using the smart hospital app**	
Yes	40
No	0
**Age (years)**	
26-30	1
31-35	5
36-40	4
41-45	5
46-50	7
51-55	9
51-60	4
61-65	3
66-70	2
**Sex**	
Female	40
Male	0
**Education level**	
Illiteracy	2
Primary school	11
High school	13
College or above	14

Note: To improve representativeness of the interviewees, objective sampling was used, and factors such as age, education level, and duration of using the app were comprehensively considered, and diverse interviewees were included.

### 2.2 Research methods

#### 2.2.1 Formulation of the interview outline

The interview outline for this study was crafted based on theoretical frameworks and methodologies. Among the many definitions of user experience, we selected the definition provided by Hassenzahl and Tractinsky [6] as it aligns with our analytical objectives: user experience is the outcome of the user's internal state (predispositions, expectations, needs, motivation, mood, etc.), characteristics of the designed system (e.g., complexity, purpose, usability, and functionality), and context in which the interaction occurs (e.g., organizational/social setting, meaning of the activity, and voluntary use). Building on this theoretical foundation, the researchers reviewed relevant literature [[7], [8], [9], [10]] and, after discussions with project team members, drafted the interview questions. After conducting pilot interviews with three participants, the final interview outline was established: (1) How did you learn about and log into the smart hospital app? (2) Do you find the smart hospital app easy to use? What are your opinions? (3) Besides our hospital's smart app, have you used other hospitals' apps? How was your experience? (4) While using the app, which interface design features of the smart hospital captured your attention? (5) Do you have any concerns when using the smart hospital app? (6) Would you recommend the smart hospital app to your patients or friends? Please explain why. (7) Do you have any other suggestions?

#### 2.2.2 Data collection

This study employed an interview research method and gathered data through semi-structured, one-on-one, in-depth interviews until data saturation was reached without the emergence of new topics. The interviewer was one of the researchers of this study, with 10 years of breast tumor care experience, was trained in qualitative interviewing, and published two core journal articles on qualitative research. The interviewer explained the purpose, methodology, and interview process of this study to the participants. Upon obtaining their informed consent, consent forms were signed, and interview times were scheduled with the respondents. The interviews were conducted in the patient conversation room of the ward, which provided a quiet and comfortable environment. All the interviews were recorded, with interview times ranging from approximately 20 to 40 min. The interview process followed the interview outline, and questioning techniques and methods were adjusted according to the participants' situations. Non-verbal behaviors, such as the participants' emotions, expressions, and body movements, were observed and recorded. Ambiguous content was promptly followed up with questions, paraphrasing, and clarification, linguistic neutrality was maintained, and respondents were encouraged to express their true feelings. After the interview ended, field notes were immediately written based on memory, including details of the interview situation, events during the interview, impressions of the respondents, and their personalities.

#### 2.2.3 Data analysis

Data were subject to interpretative phenomenological analysis (IPA), including a rigorous three-part process: naive understanding, structural analysis, and comprehensive understanding and reflection. A journal was kept, and an interview was conducted with the supervisor and health professional colleagues. This reflexivity gave the interpretation process credibility and transparency and aided in identifying potentially damaging preconceptions or bias [11]. As with the nature of interpretive phenomenology, the chosen approach was influenced by the researcher's experiences, values, and beliefs and there were multiple socially constructed realities experienced differently by different people and influenced by context. The elements of the research compliment each other in clear consensus; the interpretive phenomenological paradigm that frames the research question, the sampling and analysis methodology and the researchers own ideals. The novice qualitative researcher used several published guides and checklists to ensure the methods used were sound and thorough.

#### 2.2.4 Role of the funding source

The funder of the study had no role in the study design, data collection, data analysis, data interpretation, or writing of the study. The corresponding author had full access to all the data in the study and had final responsibility for the decision to submit for publication.

## 3 Results

### 3.1 Theme one: Positive experiences with using the smart hospital app

Most participants indicated that the smart hospital app offered a wide range of patient-centered online medical services, primarily manifested in two main areas. First, the Internet was integrated into medical services, including automated payment systems, test result inquiry devices, online admission and discharge services, and mobile consultation tools. This allowed patients to register and receive consultations anytime and anywhere and effectively saved time and space. "*Quick treatment significantly alleviates our stress*" (P13). "*Long waits and exhausting trips back and forth are physically draining*" (P6). "*Family members often have to take time off work to accompany us, which can be frustrating*" (P3).

Second, the "smart follow-up + post-discharge guidance" utilized Internet hospitals and online clinics to facilitate text and image consultations and follow-up on patient conditions, enabling online diagnosis and health education at any time. "*After being discharged from chemotherapy, unexpected situations can cause great anxiety*" (P22). "*I've experienced fever, dizziness, and vomiting. Through online consultation, I can contact my attending doctor for help, which puts me at ease*" (P15). Almost all the participants noted that the most obvious benefits were saving time and effort, convenience, and practicality, consistent with the findings of Anna Zeller et al. [12].

### 3.2 Theme two: Challenges in data sharing across multiple medical institutions

Currently, data sharing between hospitals in China remains underdeveloped, which limits resource integration and patient convenience. Additionally, the sheer volume and fragmentation of data make data maintenance time-consuming and labor-intensive, with low standardization. Multi-campus data integration systems are not fully implemented, hindering remote work [13]. Finding top hospitals and doctors is a common healthcare demand. Influenced by the "comparison shopping" mindset, people often seek consultations at multiple hospitals during the treatment of serious illnesses like cancer. However, during the treatment process, patients frequently encounter issues such as missing examination reports, incomplete treatment information, and incomplete medical records. The same tests may need to be redone due to improper report storage, increasing the cost of healthcare. "*The doctor asked for information on my radiotherapy dosage and frequency from a year ago, which was done at another hospital. My family had to visit four different hospitals to find that radiotherapy record*" (P17). " *With all the test forms, reports, and films, we don't know what we need and what we don't, so we have to carry all the examination reports every time*" (P8). "*I lost my examination reports from other hospitals and they weren't available electronically. Retesting is both costly and time-consuming, affecting my treatment*" (P29).

### 3.3 Theme three: Interpersonal communication and coping

During treatment, patients often experience heightened sensitivity and need empathetic, attentive care from healthcare providers. Most participants in this study expressed their need for assistance and support from medical staff during smart healthcare experiences. However, they found it challenging for healthcare providers to take time for detailed, repeated guidance, leading to issues such as delayed communication, information asymmetry, and communication barriers. "*I feel I need more attention from the nurses; I don't have family, and using a smartphone is too difficult for me*" (P34). "*Before chemotherapy, I wanted to know my test results as soon as possible, but doctors and nurses are too busy. I feel like I'm bothering them if I interrupt their work for this*" (P28). "*If I could check my blood test results in the app, I would feel more at ease, without worrying about being unable to undergo chemotherapy due to low white blood cell counts*" (P33). "*I often ask for help from fellow patients in the same room*" (P40). Some participants mentioned that because patients had similar experiences, they preferred communicating and sharing with each other, which made them feel relaxed and comfortable, as participant P40 noted. However, patient-to-patient communication can sometimes lead to transmission of negative or incorrect information. "*I asked a fellow patient to help me register, but she registered me at a different*

*campus, and I only found out on the day of the appointment*" (P21).

### 3.4 Theme four: Smart healthcare is not a free choice

Although all the interviewees owned smartphones, only over half used them for more than just calls and WeChat. Elderly and illiterate patients said they primarily used phones for answering calls and watching short videos. They perceived using smart hospital apps not as a free choice but rather as something they had to do due to reduced availability or closure of manual service windows in hospitals. They recognized digital services as the future trend and acknowledged the convenience brought by smart hospitals but worried about missing out on some services due to their lack of proficiency with smart technologies. This supports Christian Gybel Jensen et al.'s views [14]. Additionally, international studies indicate age differences in attitudes toward digital technology, with older adults often being less willing to use it [15]. "*My son bought me a smartphone to make it easier for me to register and see a doctor, but I still can't use it, just for calls. The smart hospital functions are great, and the nurse taught me, but I often forget where to tap*" (P14). "*Every time I get hospitalized, it feels like a test. Admission procedures, insurance referrals, payments, appointment bookings—I ask around while doing it. Meanwhile, young people in the same ward say it's easy. Technology advances too fast, and we older folks can't keep up*" (P38).

### 3.5 Theme five: Expectations for smart hospital development

#### 3.5.1 Sub-theme 1: Precise information push mechanism

All the participants recognized the construction of smart hospitals and shared their suggestions and expectations, particularly regarding the use of artificial intelligence to meet patients' diverse information needs from diagnosis to treatment and rehabilitation. Information support plays a crucial role in helping patients actively cope with their illnesses [16]. However, information transmission methods often adopt abroad-based approach, which lacks specificity and personalization. Therefore, patients may be overwhelmed by a flood of irrelevant information, making it difficult to obtain the information they truly need [17]. "*I hope the smart hospital app can push educational information to me based on my diagnosis, tailored to my needs*" (P5). "*I wish the smart hospital could develop a treatment plan based on my pathology type so that I have a general understanding of my treatment process and don't feel uncertain*" (P10).

#### 3.5.2 Sub-theme 2: Intelligent medical navigator

In recent years, AI has shown enormous potential in supporting and reshaping the medical service system and expanding and allocating quality resources, amid various factors such as national policies, economy, and technology [18]. Making smart hospitals truly intelligent involves planning treatment pathways for patients and providing voice reminders, allowing the function of an intelligent medical navigator to be realized with a smartphone. Many participants noted that hospital buildings are large and, despite the presence of numerous signs, first-time visitors often feel like they have "*entered a maze*" (P25). "*The hospital is so big, with separate north, south, east, and west zones, it's easy to get lost*" (P37). Additionally, the participants pointed out that unclear treatment steps are a major pain point during hospital visits. Feelings of confusion upon arrival and questions like "What should I do next?" were common among the participants. "*The smart hospital app should function like a GPS navigation system. When a doctor orders tests and treatments, it should immediately generate my treatment route and provide voice reminders at critical points*" (P25).

## 4 Discussion

This study identified the critical factors influencing patients' positive and negative experiences with smart hospital apps, as well as their expectations for future development. Key findings include the significance of convenience, challenges with data sharing, and the need for AI-driven personalization.

### 4.1 Summary of research findings

#### 4.1.1 Factors influencing positive experiences

Several factors influence positive patient experiences with smart hospital apps. All the participants indicated that smart hospital systems significantly reduce waiting times, enhance the efficiency of medical visits, and alleviate patients' psychological burdens. Additionally, online consultations allow patients to receive expert guidance from home and broaden access to medical care, which is particularly important for those in remote areas or with mobility issues.

Simplicity, convenience, and speed are crucial factors that promote the adoption of digital healthcare services, enabling patients to effectively manage their health and increasing their satisfaction with medical care. Moreover, smart hospital systems provide test results quickly, saving patients' time and reducing their dependence on doctors and allowing them to promptly understand their health status.

Moreover, through smart hospital apps, patients can gain a clear understanding of their medical expenses and associated charges, avoiding confusion and concern over unclear costs. This transparency enhances trust in medical services and allows patients to feel more secure when using them. Additionally, the system's automatic reminder function helps patients adhere to follow-up appointments or medication schedules, improving compliance with medical care.

In summary, smart hospital apps greatly enhance patient experiences by improving visit efficiency, expanding medical channels, providing rapid feedback, and increasing transparency. These advantages allow patients to benefit significantly from digital healthcare services, promoting better health management and driving the transformation and upgrade of healthcare services.

#### 4.1.2 Factors influencing negative experiences

Despite the effectiveness of smart hospitals in simplifying registration, payment, report inquiries, cost verification, and medical record copying processes, thereby reducing the workload for related departments, not all patient experiences have improved. Older or less educated patients often face significant challenges in using electronic technology, limiting their access to smart medical services.

Furthermore, while diverse hospital information systems enhance functionality to some extent, they result in poor data circulation. The "information silo" phenomenon prevents effective patient information sharing between hospitals, creating an information barrier that hinders smooth patient flow across different medical institutions.

With the development of smart hospitals, patients' contact with healthcare personnel has decreased. While this enhances medical efficiency, it increases feelings of loneliness and helplessness among patients. Faced with vast information systems and impersonal technology, many patients feel a lack of human care and emotional support during medical visits, prompting a desire for more face-to-face interactions with healthcare providers for psychological comfort and trust. This emotional detachment can cause anxiety when confronting health issues, thereby affecting patients’ enthusiasm for seeking medical care and health management.

Consequently, although smart hospitals have increased medical efficiency, it is essential to acknowledge these negative experiences to further optimize system design, enhance human-centered services, and ensure all patients can obtain medical services equitably and conveniently. Integrating resources, improving information-sharing mechanisms, and strengthening interactions between healthcare providers and patients can help alleviate patients' loneliness and helplessness, thereby improving their overall medical experience.

#### 4.1.3 Patient expectations for smart hospital development

Regarding future development of smart hospitals, patients hope to regain time by completing registration, examination appointments, payment, and checking appointment queues via a smartphone outside the hospital. They also expect optimized inpatient registration processes, eliminating manual personal information entry and nurse station queue registration. Additionally, with the rapid advancement of artificial intelligence, patients anticipate smarter hospitals capable of providing navigation services akin to smartphone map apps and facilitating human-machine interaction to assist vulnerable groups, such as the elderly and the less educated.

### 4.2 Reflections on the research findings

#### 4.2.1 Building smart hospitals requires more investment in human and financial resources

The knowledge system in the medical field is extraordinarily vast and complex. Medical large language models need to be "fed" extensive medical books, clinical treatment guidelines, medical papers, and real patient case data, including doctors' diagnostic records and multidimensional information, such as patients’ characteristics, test data, family history, and environmental factors [19]. Because GPT technology in healthcare is closely related to life and health, the accuracy of the output information must be exceedingly high. During extensive data training and deep learning processes, professional healthcare personnel should continually test randomly selected medical issues, verify the results generated by smart hospitals, and consistently intervene and adjust learning content and outcomes. Additionally, the use of electronic information technology is influenced by age and education level [20]. Therefore, considering this factor is crucial in the construction of smart hospitals. Medical staff should distribute leaflets, create promotional videos to guide patients, and, when necessary, provide hands-on teaching for promotion and application of the system. During use, it is vital to promptly relay patient feedback to the information department to improve information dissemination. Healthcare systems must provide timely feedback to effectively address high patient demands. Building smart hospitals requires substantial financial investment, including technology development, hardware procurement, and personnel training. AI technologies like GPT rely on large models, big data, and immense computing power and demand high server hardware configurations. The immense training tasks of large models mean that traditional CPU servers cannot support them, necessitating computing clusters composed of numerous CPU servers with stable, high-performance network connections for massive data exchange, implying significant investment costs [21]. Consequently, establishing large-scale AI computing power should rely not only on individual hospitals but also on substantial national resource investment.

#### 4.2.2 Breaking the "information wall" to promote interconnectivity in smart hospitals

Diversification of hospital information systems and poor data circulation create widespread "information silos," limiting smart healthcare within individual hospitals [22], which hinders the development of regional smart healthcare and complicates transition from informatization to smartization. Smart hospitals have advantages in optimizing medical service processes, improving service efficiency, and enhancing doctor-patient communication, breaking down barriers before, during, and after consultations with efficient pre-consultation appointments, more convenient in-consultation processes, and post-consultation intelligent follow-up [23]. Patients can manage their health by uploading photos of examination reports from different medical institutions to smart hospitals, facilitating doctor-patient review and decision-making by medical institutions [24]. Extending health services beyond hospital walls achieves a closed loop in time and space for diagnosis and treatment, realizing the convenience and efficiency of smart hospitals. Moreover, medical technology should be closely integrated with AI and big data technologies to promote the development and application of intelligent precision medicine software, aiming for high-quality medical services. Future construction of smart hospitals should not be limited to single hospitals but should rely on medical alliances or networks, leveraging new technologies to break down "walls" between hospitals and build a cloud-based collaborative platform centered on patients.

#### 4.2.3 Enhancing intelligent service capabilities of smart hospitals

Currently, smart development of public hospitals in China is still in its early stages, with local medical institutions exploring "smart management" far less than "smart healthcare" and "smart services" [25]. The unstoppable advancement of technology in the AI era will also benefit the intelligent and smart evolution of healthcare. Technologies like ChatGPT and GPT can leverage human-computer interaction interfaces, allowing the use of novel cases to generate question-and-answer tasks, forming unique narrative responses, and presenting medical information more effectively through interactive dialogue [[26], [27], [28]]. By employing technologies such as natural language processing, machine learning, and deep learning, the traditional consultation model can be thoroughly transformed, promoting the establishment of a comprehensive, integrated, and intelligent full-process medical service system covering pre-consultation, consultation, and post-consultation stages both online and offline.

**Pre-consultation:** AI appointment and triage services enable patients to communicate online from home, assisting them in the preliminary assessment of their condition through symptom descriptions, providing consultation guidance, advising on the appropriate department to visit, and recommending suitable doctors or specialists. Patients can book appointments online and receive timely notifications for hospital visits, internal navigation routes, consultation procedures, and pre-consultation precautions. Upon arriving at the hospital, AI mobile services can guide patients in taking numbers and signing in at waiting areas, with real-time updates on queue status and waiting times. While waiting, an AI mobile consultation robot simulates a doctor's thought process and conducts pre-consultation through intelligent Q&A. The system converts the patient's condition into a formally expressed chief complaint, current illness history, and medical history, aiding doctors in pre-writing electronic medical records. It analyzes and matches the symptoms and medical history described by the patient to provide preliminary diagnostic results and may suggest appropriate tests to support further medical judgment by the doctor. Based on medical knowledge bases and big medical data, GPT can construct a robust case analysis and matching system. For example, if a patient with cancer mentions experiencing fever, fatigue, and loss of appetite in recent days, GPT can preliminarily assess it as leukopenia, recommend a complete blood count test for further evaluation, and offer corresponding treatment plans and suggestions to help doctors make accurate and swift diagnostic and treatment decisions during consultations.

**During Consultation:** As the patient enters the consultation phase, the doctor has already familiarized themselves with the patient's current and past medical history, as well as the examination results, through the pre-generated electronic medical record. This process saves the doctor's time in filling out medical records, allowing them to focus more on diagnosis and treatment through observation, inquiry, and examination. The doctor only needs to adjust and refine the pre-generated electronic medical record, which significantly improves the efficiency and accuracy of medical services, reduces patient consultation time, and enhances patient experience. When prescribing medication, GPT assists by analyzing pharmaceutical theories, medical literature, and case data to remind the doctor of relevant information, such as indications, side effects, and contraindications of different drugs, aiding in medication decision-making and improving the safety and effectiveness of prescriptions, thereby enhancing the efficiency and quality of medical work.

**Post-Consultation**: The end of a consultation does not mark the end of the patient's treatment journey. AI doctors continue to accompany the patient, monitor changes in their condition, and evaluate medication use and effectiveness. Based on the patient's reported changes in condition, AI provides personalized health management plans, reasonable diet and exercise programs, and health education, acting as a health management assistant. By integrating data collected from medical-grade wearable devices on chronic disease patients—capturing continuous and comprehensive vital signs during different states (work, exercise, and sleep) —and health data maintained by users through mobile devices, information is shared and transmitted remotely. These data are archived in the hospital's patient records, and AI technologies are used to organize and analyze monitored health changes, aiding doctors in improving treatment plans, enhancing treatment levels, and establishing long-term follow-up for cancer patients. Themes of intelligent services are detailed in Table 2.

**Table 2:** Framework of intelligent service themes to enhance patient experience.

Service Node	Service Feature	Description of Intelligent Features
Pre-Consultation Services	Intelligent Triage	Utilizes AI systems with natural language processing to analyze speech and text based on symptoms and signs descried by patients, recommending suitable departments or doctors.
	Process Optimization	Redesigns and improves hospital consultation processes using AI and big data analysis to enhance the efficiency of medical resource utilization and reduce patient waiting times.
		Simplifies the consultation process.
	Self-Assessment Assistance	Employs virtual assistants or intelligent robots to help patients conduct self-assessments and preliminary screenings before consultations. Through system interactions, patients can obtain initial information and advice regarding their health status.
	Disease Prediction	Analyzes patient health data using AI technology to predict disease risks, such as identifying potential health issues early using machine learning algorithms or big data analysis.
During Consultation Services	Information Generation	Captures interactions between doctors and patients in real-time through speech recognition and natural language processing, automatically generating medical information, such as medical records and diagnostic reports.
	Diagnostic Assistance	Analyzes medical images and pathological data with AI decision support systems to provide diagnostic suggestions to doctors for more accurate clinical judgments.
	Precision Treatment	Uses AI technologies to assist in medical interventions, such as medication dosage calculations and surgical procedures, to provide more appropriate treatment plans.
	Digital Systems	Constructs a comprehensive medical management system using AI and information technology to achieve some
		"zero human" services and full-process monitoring.
Post-Consultation Services	Follow-up and Rehabilitation	Tracks and manages patient rehabilitation post-discharge using intelligent technology, with remote monitoring and data analysis to adjust rehabilitation plans in real-time.
	Health Management	Monitors and manages patients' long-term health conditions using AI technology, providing health advice, reminders, and interventions through data analysis and predictive models.

#### 4.2.4 On artificial intelligence

In recent years, artificial intelligence has achieved significant advancements in the medical field by improving medical device software and facilitating big data processing [29]. Particularly in the development of large language models and natural language processing tools like ChatGPT, application of AI is expected to become a valuable resource for future clinical practice [30]. Microsoft's Global Senior Vice President, Peter Lee, among others, described a "tri-partite model" involving doctors, patients, and machines and predicted that large language models like GPT-4 will revolutionize the healthcare industry. On February 25, 2023, the National Institute of Health and Medical Data (Shenzhen) showcased an AI product named "Hua Tuo GPT." On May 25, 2023, a domestic Internet hospital and chronic disease management platform, the Medical Consortium, released "MedGPT," the first domestically developed medical large language model based on the Transformer architecture, aiming to achieve fully intelligent diagnostic and treatment processes. Simultaneously, Google Health introduced its medical large model Med-PaLM2, which reached an "expert" level AI model after being tested in multiple clinics before its public release. Google is also exploring multimodal capabilities, such as using X-ray recognition to aid diagnosis and care. Therefore, exploring how AI technology can accurately match medical resources, create precise delivery mechanisms, and develop personalized treatment plans for patients is a challenge that medical institutions need to address in building smart hospitals.

#### 4.2.5 Research status of AI in tumor intelligent screening and risk assessment

Enhancing the dissemination of tumor knowledge is crucial for the intelligent assessment of tumor incidence risk. Currently, lightweight tumor risk intelligent assessment tools can be conveniently integrated into hospital mobile platforms like public accounts or mini-programs. These tools provide tumor screening scales for conditions such as lung nodules and lung cancer, automatically identifying high-risk patients. By intelligently generating personalized tumor screening suggestions, these tools offer guidance to high-risk groups and help improve the screening rate of high-risk tumor patients locally. Additionally, through AI large models, the system can automatically generate and push personalized tumor prevention and treatment information, enhancing public awareness of early tumor screening, diagnosis, and treatment and increasing cancer prevention and anti-cancer consciousness.

A recent study published in "Nature Medicine" created the largest standardized CT dataset for pancreatic tumors to date [31], covering 3208 real cases, training an intelligent screening model that combines plain scan CT with AI. In multi-center validations across global hospitals, this AI screening model achieved a sensitivity of 92.9 % and a specificity of 99.9 % when screening asymptomatic individuals for pancreatic cancer in check-up centers and hospitals. Another study on a breast tumor segmentation model based on dynamic contrast-enhanced magnetic resonance imaging (DCE-MRI) [32] successfully achieved segmentation of breast tumors in DCE-MRI images by creating a DCE-MRI image database for breast cancer. This study designed a tumor sensitivity synthesis module combined with a segmentation loss function, significantly improving the accuracy of tumor edge identification. On the test dataset, the model's Dice similarity coefficient reached 0.78. Moreover, AI technology can automatically perform BI-RADS scoring, assisting doctors in making quick and accurate diagnoses, and automatically generate structured text and image reports. These technological applications hold immense value for the early detection and diagnosis of breast cancer.

## 5 Clinical practice

Smart hospital apps play a crucial role in clinical practice and significantly enhance patient experience and medical efficiency. By streamlining processes such as registration, appointment scheduling, payments, report inquiries, and medical record copying, these apps enable patients to access healthcare services more conveniently, reducing waiting times and cumbersome procedures within hospitals. This is particularly beneficial for patients residing in remote areas, as telemedicine features provide the convenience of online consultations, allowing them easy access to professional medical guidance. Additionally, patients can check medical expenses and examination results in real-time, boosting trust in healthcare services and transparency in decision-making. Smart hospital apps also assist patients in managing their personal health data, promoting effective health monitoring and follow-up care. Although factors such as age, education level, and medical information security may impact the adoption of these technologies, these digital services are driving the transformation and upgrading of healthcare services, enabling patients to access the medical resources they need more efficiently and conveniently. In summary, smart hospital apps not only improve the efficiency of medical visits but also provide a more personalized healthcare experience, marking further progress toward the digitalization and intelligent evolution of healthcare services.

### 5.1 Study limitations

Our study had several limitations. First, only 40 patients with breast cancer were interviewed; possible selection bias might exist in the qualitative study. Second, the study was limited to the breast tumor department of a tertiary hospital in Wuhan. In the future, a multi-center investigation combining qualitative and quantitative research methods should be conducted to further understand patients' expectations regarding smart hospital development, providing valuable insights and guidance for researchers.

## 6 Conclusion

In this study, through qualitative interviews with 40 patients with breast cancer who are using the smart hospital app, we attempted to understand in depth patient experience with using the smart hospital app and their expectations for future construction of smart hospitals. We found that patients had diversified information needs throughout the diagnosis and treatment process, from diagnosis and treatment to rehabilitation. Information support is crucial in helping patients manage their conditions effectively. Moreover, we found deficiencies and obstacles in the construction of smart hospitals, such as “information island,” information security, single service function, and lack of intelligence. Therefore, this study holds significant implications for the future direction of smart hospital development.

## CRediT authorship contribution statement

**Xin Peng:** Writing – review & editing, Writing – original draft, Supervision, Project administration, Data curation. **Lingling Tang:** Writing – review & editing, Writing – original draft, Data curation, Conceptualization. **Ping Gao:** Writing – review & editing, Methodology, Investigation, Formal analysis, Data curation, Conceptualization. **Wei Liu:** Writing – review & editing, Validation, Supervision, Software, Funding acquisition, Formal analysis, Data curation.

## Ethical approval

This study has been approved by the Ethics Committee of Drug Clinical Trials of Huazhong University of Science and Technology. It has been carried out in the city of Wuhan, located in the middle south of China, with the registration number 20230960. The participants who have been involved in this study have signed the informed consent form before being included in the study.

## Consent for publication

Not applicable.

## Availability of data and materials

The data being used and analyzed during the current study are available from the corresponding authors upon reasonable request.

## Preprint declaration

This manuscript has been previously published as a preprint (arXiv 834035) with The Lancet on SSRN on May 23, 2024. The current submission represents an updated version of the original preprint.

## Role of the funding source

The funder of the study had no role in study design, data collection, data analysis, data interpretation, or writing of the report. The corresponding author had full access to all the data in the study and had final responsibility for the decision to submit for publication.

## Declaration of competing interest

The authors declare that they have no known competing financial interests or personal relationships that could have appeared to influence the work reported in this paper.
